The article "General Surgery Clinical Information Management System Based on Intelligent Data Management" was retracted in 2023. Reasons: signs of a paper mill; suspected computer-generated content; unreliable results or conclusions; concerns about the data.

# General Surgery Clinical Information Management System Based on Intelligent Data Management

**DOI:** 10.1155/2022/8601164

**Published:** 2022-08-01

**Authors:** Juexing Xie, Wen Luo

**Affiliations:** Zhejiang Taizhou First People's Hospital, Taizhou 318000, China

## Abstract

In order to improve the effect of surgical clinical information management, this paper combines the intelligent data management technology to construct the general surgery clinical information management system. Based on the design and development of general surgery clinical medical case information management system, this paper studies the mutual conversion between XML data and relational data, and designs a clinical medical case information management system based on the design idea of layered architecture. The clinical medical case information management system mainly adopts the modular design idea and adopts a digital microscopic image storage mode based on HDFS architecture. After building the system function structure, the system effect is verified by simulation test. From the experimental statistical results, it can be seen that the general surgery clinical information management system based on intelligent data management proposed in this paper has a good effect.

## 1. Introduction

With the advancement of medical technology and the continuous improvement of people's benchmarks for medical needs, the management of hospitals at all levels has become more complex and difficult, and the scientific requirements and standards of hospital management have also been continuously improved. Therefore, if only relying on the personal work experience of managers or the traditional manual management methods, it is far from meeting the needs of the modern medical industry. The long-term direction of the hospital in the information construction project management is to first clarify the scope of the project in the information construction. Secondly, it is necessary to ensure including cost control, improving use efficiency, and ensuring quality and quantity, and finally complete the project task objectives. In the process of project implementation, there must be necessary clear and reasonable risk assessment and risk control measures. Moreover, the construction of hospital informatization can greatly promote the management level and work efficiency of the hospital, and enhance the core competitiveness of the modern hospital. The construction of the hospital's information system is the most effective way for hospitals at all levels in China to strengthen fine management and information management, and take the road of high-precision development. At the same time, the information construction based on the computer network has promoted the scientific and standardized hospital management, which has become an important symbol to measure whether a hospital has a good social image and advanced management level. As we all know, advanced equipment is the strong and effective support needed by the medical and health service industry. Therefore, modern hospital informatization construction management also requires equipment with relatively high performance and relatively low consumption cost, which is the premise to ensure its realization. At present, the high-end medical information management technology used in the medical service industry is based on the use of a large number of instruments and equipment with computer network functions and physical health detection of patients with digital medical diagnosis and treatment.

The article "General Surgery Clinical Information Management System Based on Intelligent Data Management" was retracted in 2023. Reasons: signs of a paper mill; suspected computer-generated content; unreliable results or conclusions; concerns about the data.

Information-based medical diagnosis and treatment equipment are based on microelectronics technology, software application technology, and high-precision microprocessor technology. This is also in this era of information construction using computer networks. A remarkable achievement under the trend of development has been reached. The equipment in the medical service industry under computer intelligence is widely used, focusing on the fields of clinical data collection and processing, the fields that require online monitoring and warning of abnormal patient information, and the health sector that requires large-scale data analysis. From the hardware perspective, the large-scale microelectronic circuit integration technology is the core of the hardware. From the software perspective, the algorithm of ultra-high-speed digital signals and the very mature arithmetic processing program are the basis of the software, and these are intelligent common features of equipment. At the same time, these devices can be based on advanced wireless network communication technology and Internet technology to complete the interconnection with medical diagnosis and treatment equipment in other medical service industries, and realize the sharing of medical resources in a large area with high reliability and low cost. And the rapid development of Internet of Things technology has played a leading role in this regard. The development of my country's medical and health services and the improvement of people's living standards are inseparable from the development and progress of medical information construction. With the diversification of data processing applications, mainstream database systems continue to innovate new data models and processing algorithms, such as data warehouse and intelligent data analysis, multi-dimensional online data analysis technology and mining, and other technologies, all of which have important applications in the medical and health field.

The article "General Surgery Clinical Information Management System Based on Intelligent Data Management" was retracted in 2023. Reasons: signs of a paper mill; suspected computer-generated content; unreliable results or conclusions; concerns about the data.

The clinical medical services in the ward can be standardized through the clinical information system. We take the diagnosis and treatment information obtained by the clinical medical staff of the hospital for the diagnosis of the patient and scientifically make it specific and sequenced through a certain method, so as to obtain the best diagnosis and treatment plan, which is called the clinical path. Based on the implementation and application of the clinical information management system, the clinical path will become more standardized, which will be of great help in improving the level of medical management and the quality and efficiency of medical work. The clinical information management system enables each ward to refine and decompose the content of patients' visits by monitoring them, optimizes the quality problems of the smallest unit, and establishes a medical model that can be controlled in real time. The knowledge and management methods of the medical system can be enhanced through the clinical information management system of the ward. The ward clinical information management system is a knowledge converter of the medical system. It can transform the medical expert knowledge at the operational level into clear explicit knowledge, transform easily lost knowledge and nonsystematic knowledge into systematic knowledge assets, and at the same time help. The accumulation and integration of clinical wards into medical knowledge resources will help improve the hospital's own medical level.

This paper combines the intelligent data management technology to build a general surgery clinical information management system to improve the operation efficiency of general surgery and improve the patient experience.

## 2. Related Work

The hospital information system is a system that uses computers and communication equipment to collect, process, store, manage, retrieve, and transmit various data, materials, and other information in the hospital [1]. At present, the functional modules of the hospital information system mainly include the inpatient management module, the pharmacy management module, the outpatient diagnosis and treatment management module, the drug storehouse management module, the dean query module, the electronic prescription module, the material management module, the media management module, etc. The hospital information management system aims at providing stronger guarantees [2]. The main functions that the system can realize are doctor's visit, query function, hospitalization information, data setting and system management, and other basic functions. Among them, in the aspect of clinical information construction, the resident doctor's work module and the nurse's work module in the hospital information system are particularly important. The resident doctor's work module mainly realizes the functions of the clinician in the hospital to write the patient's condition, take daily routine medical orders, and inquire about the various examinations of the inpatient; the work module of the ward nurse provides the management of medical orders in each inpatient ward bed management, hospitalization status of patients, and printing various types of doctor's orders, checklists, and other items [3]. A system that uses electronic equipment based on integrated circuit technology to save, manage, transmit, and reproduce patient medical records is called electronic medical records. The clinical information management system of the ward is based on the two major medical information systems of the hospital information system and the electronic medical record [4]. It obtains the effective information of the patients, integrates it, and displays it on the electronic screen interface, replacing the traditional manual transcription mode of the nurses in the ward [5].

The article "General Surgery Clinical Information Management System Based on Intelligent Data Management" was retracted in 2023. Reasons: signs of a paper mill; suspected computer-generated content; unreliable results or conclusions; concerns about the data.

The hospital information management system, abbreviated HIS, is a system that includes all aspects of the hospital's work and provides a full range of information security for the entire medical process. Management information system, clinical medical information system, and regional medical information network are three stages of hospital information system [6]. The hospital information system proposes three major systems: the hospital information system data model, the hospital information system data management model, and the hospital information system data application model from the aspects of technology, management, and business application, which are closely related to each other. HIS design includes subsystem functional structure design, database design, and program development [7]. The HIS system is mainly constructed and designed based on the hospital information data application system, the hospital information data host system, the hospital information data network system, and the hospital information data physical environment. Relying on the integration of data and business, it finds a new way for cooperation. Usually, the hospital information system consists of hospital management system, outpatient management system, medical technology management system, inpatient management system, etc. These subsystems together build the hospital information system. Each subsystem has a corresponding functional module framework. The core part of the hospital information system is the database, which is the basic core of the HIS system. The more commonly used databases are Oracle and SQL Server [8].

The article "General Surgery Clinical Information Management System Based on Intelligent Data Management" was retracted in 2023. Reasons: signs of a paper mill; suspected computer-generated content; unreliable results or conclusions; concerns about the data.

A large amount of important medical-related information in the hospital is stored in the electronic medical record system in electronic form [9]. Its content includes all the information of a paper medical record. In the basic technical architecture of the system, WebService is used, which is mainly implemented on the NET platform. The electronic medical record is based on the intelligent input module of XML technology and makes full use of the advantages of XML technology to realize the input mode of effective combination of free text input and form input [10]. It can easily store XML documents into Oracle database and can effectively convert relational databases and XML documents. Based on such conditions, XML can easily realize the query function, has the ability to perform poststructural analysis of text information, can quickly convert text information into data elements, making it convenient for computer statistics, and can be shared and meet the requirements of the Ministry of Health [11]. The electronic medical record system has specialized data integration middleware and open software architecture, which can make the originally complicated and massive data integration work simple and smooth [12]. At the same time, for the docking of hospital information system, inspection system, and medical imaging system, it can be completed by editing the corresponding configuration file. This docking method no longer requires any extra code-level modification. Read-only data integration is usually completed within 2–3 days [13]. The network communication framework of the medical service industry based on TCP/IP technology is the basis for ensuring the electronic medical record system. The core of this framework is to guarantee a complete medical information service. Through this core service, the system connection and integration between hospitals are possible. The ultimate purpose of this method is to change the traditional way of clinical medical work and process coordination, and to provide an active, real-time, and collaborative information exchange platform [14].

## 3. General Surgery Clinical Information Management System Based on Intelligent Data Management

The basic building blocks of an information model include entities, entity attributes, and relationships between entities. Among them, the entities are a collection of abstract things or reality with the same characteristics, which is divided into independent entities and subordinate entities. Attributes are the characteristics or properties of entities, and inter-entity relations refer to the logical relationships that exist between entities. This design is to establish an information model according to the business flowchart, in order to sort out the types of information that need to be coded, and to provide the basis for the business logic relationship for the design of the operating mode of the system. The key to the entire information system is how to realize the transmission and storage of the entire information, as well as the processing of changes. The entity set of the information model is established according to the clinical pathway admission assessment flowchart, as shown in Figure 1.

The article "General Surgery Clinical Information Management System Based on Intelligent Data Management" was retracted in 2023. Reasons: signs of a paper mill; suspected computer-generated content; unreliable results or conclusions; concerns about the data.

Figure 1 shows an information model diagram of path admission evaluation. Among them, entities are divided into independent entities and subordinate entities, entities have certain attributes, and there is an attribute that uniquely identifies each instance, that is, a number. The primary key of the dependent entity inherits the independent entity as one of its own attributes, which is used to indicate which independent entity is the child entity. In the information model of path admission assessment, independent entities include patients, visiting departments, registration offices, auxiliary departments, and clinical paths to which they belong. In addition, other entities exist because of the existence of independent entities, such as the registration form attached to the patient and the registration office department number. In this information model, the logical relationship between the registration office and the registration form is that the registration office writes the registration form, and there is a one-to-many correspondence, which reflects the connection between the two entities. Second, there is a one-to-one correspondence between patients and registration slips, and all of this information can be reflected in the information model. It is precisely because of the existence of such a logical relationship between these entities that the information carrier can successfully transmit the target to the entity that needs the target. The design of this model reflects the goals and attributes in the path admission process, and provides a basis for the design of the database [15].

An important part of the regional pathological information management system is the remote pathological consultation system. One of the main goals of its design is to solve the problem of unbalanced pathological resources in the region. Due to the limitations of pathological levels in different regions, some hospitals do not have the technology to solve difficult cases, so it is necessary to initiate consultation requests to higher-level hospitals. After receiving consultation in a higher-level hospital, patients or hospitals are often required to send specimens or slides to the higher-level hospital, which greatly increases the cost of medical treatment in some remote areas. On the other hand, there are many patients in large hospitals, the workload of doctors is heavy, and pathological examinations often need to wait for a long time, which is likely to miss the best time for diagnosis. The remote pathological consultation system realizes the remote transmission of pathological information through modern medical information technology and realizes long-distance pathological consultation. It not only overcomes geographical barriers and greatly reduces the time for pathological examination and diagnosis, but also makes communication between the same industry more closely through Internet technology. This promotes the medical re-education of pathology, thereby improving the uneven distribution of pathological resources and realizing the sharing of pathological resources. Pathological consultation mainly uses the digital slide scanning system to stitch the slide scans under the digital microscope into full-field pathological slide images (digital slides). After a lower-level doctor initiates a consultation, the patient information and digital slice information can be uploaded to the system, and the higher-level doctor will send back the results after consultation based on the received patient information and digital slice information. The remote pathological consultation system based on the B/S development model can complete a diagnosis by logging into the system in the network environment through a tablet computer, mobile phone, or computer.  Figure 2 shows a flowchart of a consultation initiated by a subordinate pathologist based on the regional pathological information management system [16].

The article "General Surgery Clinical Information Management System Based on Intelligent Data Management" was retracted in 2023. Reasons: signs of a paper mill; suspected computer-generated content; unreliable results or conclusions; concerns about the data.

The metadata server NameNode of HDFS is responsible for managing the system namespace and user access to files. When a user writes a file, it waits until the file data size reaches one block before contacting the metadata server. Then, the metadata server stores the file obituary information in its namespace, assigns a block to the file, and returns the ID of the DataNode where the block is located to the client. The NameNode node server stores the two most important tables in the entire system: the mapping between the file name and the block sequence and the mapping between the data block and the machine list. The filename and block sequence mapping stores the namespace of the entire file system directory, and the mapping between data blocks and machine lists is the correspondence between a single data block-9 machine list. Through these two mappings, the client can find the DataNode where the block is located according to the directory information stored in the NameNode. The DataNode deployed on the PC is responsible for the operation and management of its own stored data. The default block size of HDFS is 64 MB. If a large number of small data files are stored in the HDFS file system, the metadata node NameNode will consume too much memory and reduce the performance of the entire HDFS cluster. Therefore, HDFS is optimized for the storage of large data files above PB level. In the pathological consultation system, digital microscopic images often reach hundreds of GB of data, and such a large amount of data requires a storage solution specially designed for massive data. To solve this problem, we adopt a digital microscopic image storage mode based on HDFS architecture, as shown in Figure 3.

The system function modules of the clinical medical case information management system include six modules: data integration, document management, template configuration, case retrieval, statistical analysis, and public interface. The functions and relationships of these six modules in the application are as follows. First, the system extracts the corresponding data from the relational database SQL Server through the data integration function and converts it into data that conforms to the XML format specification. Then, the data are entered into the XML database, and the functions related to the data query of the system, such as document viewing, case retrieval, statistical analysis, and other functions, can be used for the next data query and statistical operation. Among them, the data display style of the document viewing function module needs to be configured with the template configuration function module first, and the XSLT file content is used to configure the display mode, such as horizontal version and vertical version. The structure of the whole system is shown in Figure 4. Its relationship with other systems is shown in Figure 5 [17].

There are two paths for converting relational data to XML data. First, every time the data are queried from the relational database, it is immediately imported into the XML database. Second, all the data in the relational database are queried out, converted into XML data, and then imported into the XML database. The advantage of the first method is seamless connection, but it will delay the time of data integration of the whole system. If an error occurs in the middle of this behavior, the XML database will have to perform a large number of rollback operations, and it is difficult to guarantee the accuracy of the data and the stability of the system. The second way is to first convert the relational database data into XML data and store it in the hard disk, and then read the XML data from the hard disk and store it in the XML database. This will produce XML data that take up hard disk space and take time to read and write to the hard disk, and the overall time will be a little more than the first method. Then, because the process of exporting and importing data from the relational database to the XML database is separate, if there is a problem in the export process, the data in the XML database may not be affected. Therefore, the system adopts the second data integration method, and the data integration management module architecture is shown in Figure 6 [18].

The article "General Surgery Clinical Information Management System Based on Intelligent Data Management" was retracted in 2023. Reasons: signs of a paper mill; suspected computer-generated content; unreliable results or conclusions; concerns about the data.

The BaseDao layer calls the XMLConfigClientTemplate class that encapsulates the read database operation statement, and when there is a return result, encapsulate the returned result in a corresponding list or a single object to interact with the database. The function of the XMLConfigClientTemplate class to read the database operation statement is to call the XMLConfigUtil class to read the database operation statement from the database query statement configuration file. In order to realize the independence of database operation statements from Java programs as much as possible, the system places database operation statements in several separate configuration files. Programmers only need to write static operation statements and required dynamic parameters in the configuration file and specify the values of the dynamic parameters in the Java program, and then the XMLConfigUtil class parses and generates the corresponding database operation statements. The operation on the database is to obtain the database session by calling the get XQSession method of the DptXMLDBSessionFactory class. Then, by calling the database operation method given by it, the generated database operation statement is passed in to perform the database operation. The operation of encapsulating the returned result in the corresponding list or single object is to parse the returned result into the corresponding class or list through the function provided by XML Operate. Its function implementation class call structure is shown in Figure 7.

## 4. Effect Verification of General Surgery Clinical Information Management System Based on Intelligent Data Management

After the system is constructed, the system of this paper is constructed on the MATLAB platform. This paper collects various types of information from hospitals as input and starts from the aspects of clinical information collection, clinical information processing, clinical information transmission, and user experience in the system to test the general surgery clinical information management system based on intelligent data management proposed in this paper. The statistical test results are shown in Table 1–4.

The article "General Surgery Clinical Information Management System Based on Intelligent Data Management" was retracted in 2023. Reasons: signs of a paper mill; suspected computer-generated content; unreliable results or conclusions; concerns about the data.

From the statistical results of the above experiments, it can be seen that the general surgery clinical information management system based on intelligent data management proposed in this paper has a good effect, so it can be applied to the clinical practice of general surgery.

## 5. Conclusion

The clinical medical case information management system is a platform for efficient storage and processing of unstructured data for information systems. It can use a tree structure to organize various data including multimedia resources required by the website. Moreover, the construction and implementation of the clinical medical case information management system will be able to solve the problems of query, storage, and insertion of different unstructured data. In addition, it provides perfect data processing services for the application systems connected to the system, thereby solving the problem that unstructured data cannot be efficiently processed. The clinical medical case information management system mainly uses the powerful processing function of XML database for unstructured data to solve the problem that enterprise unstructured data are difficult to efficiently integrate into the information system, resulting in insufficient overall processing of enterprise data, so that all data can be uniformly and efficiently processed in the information system. This article combines the intelligent data management technology to construct the general surgery clinical information management system. From the experimental statistical results, it can be seen that the general surgery clinical information management system based on intelligent data management proposed in this paper has a good effect.

## Figures and Tables

**Figure 1:** Path admission evaluation information model.

**Figure 2:** Flowchart of consultation in regional pathological information management system.

**Figure 3:** HDFS-based digital microscope image storage mode.

**Figure 4:** Structure diagram of system functions.

**Figure 5:** The relationship diagram between the clinical medical case information management system and other systems.

**Figure 6:** Architecture diagram of the data integration module.

**Figure 7:** Structure diagram of class call.

**Table 1:** Information collection effect of general surgery clinical information management system.

Number	Information collect	Number	Information collect	Number	Information collect	Number	Information collect
1	91.23	23	84.62	45	88.39	67	93.44
2	87.50	24	91.37	46	87.82	68	85.15
3	88.99	25	84.23	47	86.03	69	86.74
4	93.50	26	84.36	48	87.39	70	91.95
5	90.56	27	89.68	49	90.82	71	91.02
6	90.84	28	85.51	50	84.26	72	91.47
7	85.07	29	88.83	51	87.09	73	91.15
8	85.71	30	88.61	52	93.01	74	84.53
9	87.84	31	89.29	53	84.69	75	91.91
10	91.63	32	87.23	54	92.48	76	85.37
11	86.37	33	87.00	55	84.82	77	92.67
12	87.12	34	90.00	56	87.74	78	84.78
13	91.12	35	84.83	57	87.51	79	89.49
14	87.74	36	93.39	58	91.06	80	85.07
15	85.38	37	89.92	59	92.81	81	91.85
16	87.35	38	84.07	60	87.90	82	87.47
17	88.89	39	85.31	61	89.73	83	84.25
18	89.21	40	91.90	62	88.10	84	87.86
19	86.93	41	89.50	63	87.90	85	93.69
20	91.21	42	86.61	64	86.74	86	84.08
21	93.67	43	89.85	65	91.44	87	93.23
22	85.18	44	89.41	66	84.39	88	85.13

The article "General Surgery Clinical Information Management System Based on Intelligent Data Management" was retracted in 2023. Reasons: signs of a paper mill; suspected computer-generated content; unreliable results or conclusions; concerns about the data.

**Table 2:** Information processing effect of general surgery clinical information management system.

Number	Information processing	Number	Information processing	Number	Information processing	Number	Information processing
1	84.73	23	86.78	45	91.65	67	85.37
2	86.99	24	84.80	46	88.41	68	89.89
3	89.28	25	93.43	47	91.84	69	87.57
4	84.41	26	87.93	48	85.42	70	93.91
5	91.22	27	86.11	49	93.31	71	93.02
6	91.50	28	93.17	50	84.94	72	91.34
7	85.22	29	87.37	51	92.83	73	90.36
8	89.01	30	91.67	52	85.49	74	87.79
9	89.18	31	84.48	53	93.69	75	92.07
10	86.06	32	93.86	54	91.30	76	93.21
11	86.37	33	89.51	55	84.31	77	92.72
12	85.49	34	93.26	56	90.28	78	90.82
13	88.13	35	93.05	57	93.47	79	88.11
14	88.69	36	89.11	58	93.64	80	89.45
15	91.00	37	84.39	59	87.63	81	91.14
16	88.39	38	93.94	60	90.68	82	89.41
17	85.44	39	91.91	61	92.09	83	88.70
18	87.08	40	93.28	62	88.90	84	85.13
19	92.84	41	92.79	63	92.50	85	91.28
20	84.24	42	89.72	64	93.99	86	88.55
21	85.43	43	93.43	65	88.12	87	90.83
22	91.63	44	87.52	66	88.29	88	88.05

**Table 3:** Information transmission effect of general surgery clinical information management system.

Number	Information transfer	Number	Information transfer	Number	Information transfer	Number	Information transfer
1	91.78	23	86.57	45	86.27	67	84.12
2	87.68	24	91.51	46	91.29	68	90.98
3	90.86	25	89.75	47	84.79	69	91.58
4	87.82	26	92.65	48	88.95	70	89.05
5	89.25	27	93.08	49	93.43	71	87.81
6	86.91	28	89.15	50	87.57	72	90.47
7	89.86	29	86.55	51	93.24	73	88.40
8	91.08	30	92.06	52	88.21	74	93.93
9	85.87	31	88.68	53	90.84	75	93.89
10	87.20	32	91.90	54	85.39	76	85.72
11	86.84	33	90.06	55	88.06	77	87.34
12	88.37	34	93.30	56	87.71	78	89.66
13	87.89	35	91.99	57	92.92	79	84.40
14	92.01	36	87.83	58	86.06	80	86.97
15	92.11	37	92.57	59	93.39	81	87.12
16	85.86	38	93.97	60	90.59	82	84.03
17	84.27	39	93.59	61	90.25	83	93.23
18	89.63	40	92.34	62	84.43	84	86.01
19	91.59	41	86.59	63	91.05	85	84.81
20	84.66	42	91.46	64	89.58	86	85.08
21	86.05	43	91.56	65	87.15	87	92.56
22	87.94	44	90.10	66	93.55	88	93.35

The article "General Surgery Clinical Information Management System Based on Intelligent Data Management" was retracted in 2023. Reasons: signs of a paper mill; suspected computer-generated content; unreliable results or conclusions; concerns about the data.

**Table 4:** User experience of general surgery clinical information management system.

Number	User experience	Number	User experience	Number	User experience	Number	User experience
1	93.70	23	85.01	45	86.24	67	85.27
2	87.26	24	90.35	46	84.64	68	89.29
3	84.82	25	86.07	47	88.32	69	90.62
4	86.13	26	91.66	48	87.07	70	85.96
5	89.71	27	84.43	49	88.78	71	91.45
6	90.44	28	91.94	50	89.64	72	84.57
7	88.09	29	85.96	51	93.67	73	84.71
8	93.60	30	90.27	52	88.27	74	84.95
9	84.35	31	93.17	53	91.03	75	87.61
10	92.19	32	93.51	54	93.86	76	87.32
11	93.04	33	87.16	55	90.61	77	91.44
12	90.49	34	84.93	56	85.19	78	92.80
13	86.94	35	90.61	57	93.67	79	87.76
14	84.58	36	84.97	58	84.45	80	84.60
15	84.73	37	84.24	59	84.48	81	89.74
16	90.19	38	92.69	60	93.21	82	88.55
17	87.46	39	87.72	61	90.37	83	84.70
18	89.30	40	87.95	62	85.47	84	87.26
19	88.15	41	87.64	63	86.35	85	87.34
20	84.44	42	85.86	64	84.34	86	84.27
21	89.45	43	93.26	65	89.66	87	92.60
22	86.41	44	93.42	66	90.52	88	93.15

## Data Availability

The labeled dataset used to support the findings of this study is available from the corresponding author upon request.
